The article "Forkhead box (FOX) G1 promotes hepatocellular carcinoma epithelial-Mesenchymal transition by activating Wnt signal through forming T-cell factor-4/Beta-catenin/FOXG1 complex" was retracted in 2023. Reasons: duplicated images; original data or images not available; unreliable data; lack of ethics approval or compliance.

# Forkhead box (FOX) G1 promotes hepatocellular carcinoma epithelial-Mesenchymal transition by activating Wnt signal through forming T-cell factor-4/Beta-catenin/FOXG1 complex

**DOI:** 10.1186/s13046-019-1433-3

**Published:** 2019-11-27

**Authors:** Xingrong Zheng, Jiaxin Lin, Hewei Wu, Zhishuo Mo, Yunwen Lian, Peipei Wang, Zhaoxia Hu, Zhiliang Gao, Liang Peng, Chan Xie

**Affiliations:** 1 Department of Infectious Diseases, the Third Affiliated Hospital of Sun Yat-sen University, 600# Tianhe Road, Guangzhou, 510630 Guangdong Province China; 2 Key Laboratory of Tropical Disease Control, Ministry of Education, Sun Yat-sen University, Guangzhou, 510630 Guangdong Province China; 3 Guangdong Provincial Key Laboratory of Liver Disease, Guangzhou, China

**Keywords:** FOXG1, HCC, EMT, Wnt/β-catenin

## Abstract

**Background:**

Forkhead box G1 (FOXG1) is a member of the Fox transcription factor family involved in regulation of many cancers. However, the role of FOXG1 in hepatocellular carcinogenesisis largely unclear. The present study aimed at examining the biological function and underlying mechanism of FOXG1 on hepatocellular carcinoma (HCC) tumor metastasis as well as its clinical significance.

**Methods:**

Levels of FOXG1 were determined by immunohistochemical and real-time PCR analysis in HCC cell lines and human HCC samples. The effect of FOXG1 on cancer cell invasion and metastasis was investigated in vitro and in vivo in either FOXG1-silenced or overexpressing human HCC cell lines. Immunoprecipitation and chromatin immunoprecipitation assays were performed to investigate the interaction of FOXG1, β-catenin, TCF4 and the effect on Wnt target-gene promoters.

**Results:**

In human HCC, the level of FOXG1 progressively increased from surrounding non tumorous livers to HCC, reaching the highest levels in metastatic HCC. Furthermore, expression levels of FOXG1 directly correlated with cancer cell epithelial-mesenchymal transition (EMT) phenotype. In FOXG1-overexpressing cells, FOXG1 promotes the stabilization and nuclear accumulation of β-catenin by directly binding to β-catenin and it associates with the lymphoid enhancer factor/T cell factor proteins (LEF/TCFs) on Wnt responsive enhancers (WREs) in chromatin.

**Conclusions:**

The results show that FOXG1 plays a key role in mediating cancer cell metastasis through the Wnt/β-catenin pathway in HCC cells and predicts HCC prognosis after surgery. Targeting FOXG1 may provide a new approach for therapeutic treatment in the future.

## Background

Worldwide, HCC is still a malignant tumor with high incidence and mortality, remaining a great threat to human health. According to the 2018 cancer statistics report, the five-year relative survival rate for HCC patients is only 18%. However, the mortality rate of males consistently sustain higher and continue to rise at a rate of 1.6% per year [1]. Due to the complex mechanism, every known treatment is poorly responded [2]. Abnormal Wnt signal activation caused by genetic mutationis was responsible for 30% of hepatitis B virus-(HBV)-related HCC and involved in epithelial-mesenchymal transition (EMT), which is the main mechanism of tumor metastasis [3]. Besides, aberrant Wnt/β-catenin activation has been reported in approximately 50% of all HCC [4]. Therefore, identifying alternative mechanisms and molecular factors for predicting tumor metastasis will help improve the overall clinical management of HCC patients.

The article "Forkhead box (FOX) G1 promotes hepatocellular carcinoma epithelial-Mesenchymal transition by activating Wnt signal through forming T-cell factor-4/Beta-catenin/FOXG1 complex" was retracted in 2023. Reasons: duplicated images; original data or images not available; unreliable data; lack of ethics approval or compliance.

EMT is a normal physiological process that converts epithelial cells into mesenchymal cells. However, the process is frequently exploited by cancer cells to migrate to surrounding and distant regions. Characteristics of EMT observed in the tumor progressions include the decreased intercellular adhesion, loss of epithelial markers (e.g. E-cadherin), acquisition of mesenchymal markers (including vimentin and N-cadherin), etc. [5]. These EMT related cellular alterations leading to a more mesenchymal state are often associated with poor prognosis.

A key role in the molecular pathway that promotes EMT is the Wnt/β-catenin signaling pathway [6]. When the signaling pathway activated, β-catenin begins to accumulate in the cytoplasm and translocate toward the nucleus, where it works with the TCF/LEF protein to activate the transcription of multiple target genes [7]. In the absence of Wnt, β-catenin would be degraded by the destruction complex containing APC, Axin and GSK-3β kinase, and cause transcription repression [8]. Dysregulated activation of the Wnt signaling pathway can promote the progress of EMT and the metastasis of lesions in many cancers [9, 10]. Studies have indicated that aberrant Wnt/β-catenin pathway activation in HCC promotes proliferation and sorafenib resistance [11], suggesting that hyperactivation of the Wnt/β-catenin signaling pathway contributes to tumorigenic properties and the invasive phenotype. It has been reported that CTNNB1 and AXIN activated mutations were present in 44% (40/90) of non-HBV-related HCC cases (*P* < 0.0001) [12]. Furthermore, approximately 50% of HCC cases exhibited the hyperactivation of Wnt/β-catenin signaling pathway [4]. Hence, the exploration of underlying hyperactivation of Wnt/β-catenin signaling in HCC may reveal therapeutic targets for prevention or treatment of the metastasis.

FOX transcription factor family plays an important role in the Wnt pathway [13, 14]. Besides of that, overexpression of FOXG1 increases the capacity of tumor cells to migrate and invade in vitro and promote tumor metastasis in vivo [15, 16], which predict a poor prognosis. FOXG1 can bind to DNA recognition sequences and act as a transcription suppressor along with corepressor proteins [17–19]. However, FOXG1-mediated repression is not restricted to direct DNA interaction, it also works through protein-protein interaction, independently of binding to DNA recognition sequence [20, 21]. Although preliminary understanding, the underlying mechanism of FOXG1 is still far from clear.

The article "Forkhead box (FOX) G1 promotes hepatocellular carcinoma epithelial-Mesenchymal transition by activating Wnt signal through forming T-cell factor-4/Beta-catenin/FOXG1 complex" was retracted in 2023. Reasons: duplicated images; original data or images not available; unreliable data; lack of ethics approval or compliance.

In our current study, we aimed to explore the possibility of FOXG1 as a key component of the Wnt signaling pathway regulating the nuclear accumulation of β-catenin, determine the biological interaction of FOXG1/β-catenin/TCF4 on HCC EMT and lesions metastasis, and further clarify their clinical significance. These findings suggest that FOXG1 may be a valuable prognostic factor and potential therapeutic target for HCC.

## Materials and methods

### Cell lines and culture

HCC cell lines, including HepG2, Huh7, Hep3B, PLC/PRF5y, HCCLM3, MHCC97L, and MHCC97H, were obtained from the Guangdong Provincial Key Laboratory of Liver Disease and grown in Dulbecco’s modified Eagle medium (DMEM, Invitrogen, Carlsbad, CA, USA). LO2 normal human liver cells were maintained in RPMI-1640 medium (Gibco, Grand Island, NY, USA). All medium was supplemented with 10% fetal bovine serum (FBS, HyClone, Logan, UT, USA), 2 mM L-glutamine, 100 units/ml penicillin, and 100 μg/ml streptomycin in an atmosphere of 5% CO_2_ at 37 °C.

### Patients and tumor tissues

A total of 105 paraffin-embedded, archived HCC samples that had been histopathologically and clinically diagnosed as HCC at the Sun Yat-sen University Cancer Center from 1995 to 2011 were used in the current study. Ten fresh HCC tissue samples were obtained from patients undergoing HCC resection at the Department of Hepatobiliary Surgery of the Third Affiliated Hospital of Sun Yat-sen University. Prior patient consent and approval of the Institutional Research Ethics Committee of the Third Affiliated Hospital were obtained for the use of the clinical materials described above for research purposes. The clinicopathologic characteristics of the 105 patients are summarized in Additional file 1: Table S1.

### Immunoprecipitation (IP)

Cells were lysed in co-IP buffer (10 mM HEPES [pH 8.0], 300 mM NaCl, 0.1 mM EDTA, 20% glycerol, 0.2% NP-40, and protease and phosphatase inhibitors). Lysates were centrifuged and cleared by incubation with 25 μl of Protein A/G gel for 1 h at 4 °C. The pre-cleared supernatant was subjected to IP using first antibodies at 4 °C overnight. Then, the protein complexes were collected by incubation with 30 μl Protein A/G gel for 1 h at 4 °C. The collected protein complexes were washed six times with co-IP buffer and analyzed by western blotting.

The article "Forkhead box (FOX) G1 promotes hepatocellular carcinoma epithelial-Mesenchymal transition by activating Wnt signal through forming T-cell factor-4/Beta-catenin/FOXG1 complex" was retracted in 2023. Reasons: duplicated images; original data or images not available; unreliable data; lack of ethics approval or compliance.

### Chromatin immunoprecipitation-qPCR (ChIP-qPCR) assays

For the ChIP assay, 5 × 10^6^ cells were prepared with the ChIP assay kit (Cell Signaling Technology, Danvers, MA, USA) according to the manufacturer’s instructions. DNA complexes were immunoprecipitated using the anti-FOXG1 (USBio, ABIN2668064) or anti-β-catenin (USBio, ABIN442212) or anti-TCF4 (USBio, ABIN2372673) antibodies and then eluted by incubation for 30 min at 37 °C in 100 μl of 10 mM DTT. After centrifugation, the supernatant was diluted 50× with ChIP buffer. The resulting precipitated DNA samples were further analyzed by qPCR. The primers are listed in section “RNA extraction, reverse transcription, and qPCR” in Additional file 2.

### Immunofluorescence (IF)

HCC cells, cultured on cover slips, were transfected with pcDNA3.1-FOXG1 or FOXG1 shRNA and the respective controls pcDNA-vector or nonsense siRNA control reagents for 48 h. Cells were washed, fixed in 4% paraformaldehyde for 15 min, and then rinsed in PBS three times for 5 min each, and blocked with 5% BSA in PBS for 30 min at 25 °C. Primary antibody was added and incubated for 1 h at 37 °C and then detected using FITC-conjugated secondary antibody. Images were captured using a fluorescence microscope.

### Immunohistochemistry (IHC)

We used 2-μm sections of formalin-fixed paraffin-embedded HCC tissue samples for IHC staining. All sections were treated routinely with the EnVision system (Dako, Glostrup, Denmark). The primary antibodies were anti-FOXG1 (1:80, Abcam), anti-TCF4 (1:200, Abcam), and anti-β-catenin (1:200, BD Biosciences). IHC staining results were evaluated in a double-blind manner by two experienced pathologists and are presented as the average score. The results of IHC staining were scored on a scale of 0–12. The value of the staining intensity and the percentage of positive cells were graded. It was presented as the average score for the extent of IHC staining. Scores for different groups of tissues were compared using Student’s *t*-test; *P* < 0.05 was considered significant.

### Statistical analysis

All values are presented as mean ± standard deviation (SD). Significant differences were determined using SPSS 16.0 software (SPSS, Chicago, IL, USA). Student’s *t*-test was used to determine statistical differences. The chi-square test was used to analyze the relationship between FOXG1 expression and clinical pathological characteristics. Survival curves were plotted using the Kaplan–Meier method and compared by log-rank test. *P* < 0.05 was considered significant.

The article "Forkhead box (FOX) G1 promotes hepatocellular carcinoma epithelial-Mesenchymal transition by activating Wnt signal through forming T-cell factor-4/Beta-catenin/FOXG1 complex" was retracted in 2023. Reasons: duplicated images; original data or images not available; unreliable data; lack of ethics approval or compliance.

Other experimental procedures are available in Additional file 2.

## Results

### FOXG1 was up-regulated in HCC and associated with poor prognosis

By analyzing the datasets from the GEO Publication Omnibus, we found the expression of FOXG1 was significantly up-regulated in adjacent non tumor tissue (ANT) and cirrhotic liver tissue (CIRR), with the highest level in HCC tissues (HCC) compared with healthy liver tissue (HEAL) (Fig. 1a). FOXG1 expression was up-regulated in 7 HCC cell lines compared with normal LO2 liver cells detected by qPCR and western blotting analysis (Fig. 1**b** and **c**). Furthermore, FOXG1 expression was higher in HCC with vascular invasion (Fig. 1d). Therefore, both the published datasets and our results suggest that FOXG1 is up-regulated in HCC.

**Fig. 1:** Elevated expression of FOXG1 is associated with metastasis in human HCC. **a** FOXG1 mRNA levels in hepatocellular carcinoma (HCC) tissue dataset (GSE25097). CIRR: cirrhosis tissues, HEAL: healthy liver tissues, ANT: adjacent non tumor tissues, HCC: hepatocellular carcinoma. **b** Expression of FOXG1 mRNA and (**c**) protein in LO2 normal human liver cell line (as comparison control) and the indicated cultured HCC cell lines. GAPDH was used as a loading control. **d** Western blotting analysis of FOXG1 protein in each of the non-metastatic (N) and metastatic (M) HCC tissue from ten patients. **e** Expression of FOXG1 protein in 64 non-metastatic (N) and 41 metastatic (M) HCC tissues. **f** Overall survival of patients with HCC with low vs. high FOXG1 expression. Error bars represent SD from three independent experiments. *P < 0.05

To further investigate whether up-regulated FOXG1 is involved in HCC progression, a total of 105 archived paraffin-embedded HCC specimens were subjected to qPCR and IHC staining using a human anti-FOXG1 antibody. qPCR analysis confirmed that the expression of FOXG1 in metastatic tissues was significantly higher than that in non-metastatic tissues (Fig. 1e). Statistical analysis showed that patients with high expression of FOXG1 tended to have higher TNM grades and α-fetoprotein (AFP) levels, higher probability of vascular metastasis and shorter survival time (Additional file 1: Table S2). Similarly, Kaplan-Meier survival analysis supported the higher expression of FOXG1 correlated to lower overall survival rate (Fig. 1f).

### Ectopic expression of FOXG1 augments HCC aggressiveness in vitro

To investigate the potential role of FOXG1 in EMT, we transfected Huh7 and PLC/PRF5y cells with FOXG1 expression vector to achieve stable ectopic expression of FOXG1, and control cells were transfected with control vector. The expression levels of endogenous FOXG1 in these two cell lines were relatively moderate (Fig. 1b and c). As demonstrated by Western blotting (Fig. 2a) and Immunofluorescence (Fig. 2b) analysis, ectopic FOXG1 significantly reduced the expression of E-cadherin and α-catenin, but highlighted the vimentin and fibronectin, suggesting that FOXG1 enhanced the invasiveness of HCC.

The article "Forkhead box (FOX) G1 promotes hepatocellular carcinoma epithelial-Mesenchymal transition by activating Wnt signal through forming T-cell factor-4/Beta-catenin/FOXG1 complex" was retracted in 2023. Reasons: duplicated images; original data or images not available; unreliable data; lack of ethics approval or compliance.

**Fig. 2:** Overexpression of FOXG1 promotes cell mobility and invasion by inducing epithelial-mesenchymal transition (EMT). **a** Western blotting analysis and **b** Immunofluorescence analysis of expression of epithelial cell markers (E-cadherin and α-catenin) and mesenchymal cell markers (vimentin and fibronectin) in indicated cells transfected with FOXG1 expression vector or control vector. Nuclei counterstained with DAPI. GAPDH was used as a loading control. **c** Representative migrating images of the indicated Huh7 and PLC/PRF5y cells on uncoated Transwell devices in five random fields. **d** Quantification of the invading cells of the indicated Huh7 and PLC/PRF5y cells on Matrigel-coated Transwell devices in five random fields. Values represent mean ± SD. *P < 0.05. **e** Representative micrographs of wound healing assay of the indicated Huh7 and PLC/PRF5y cells. Wound closures were photographed at 0, 24, and 36 h after wounding. All experiments were repeated at least three times with similar results

Consistent with this, Matrigel-coated (for invasion) or -uncoated (for migration) Transwell assay confirmed that overexpression of FOXG1 increased the invasiveness and migration of the PLC/PRF5yand Huh7 HCC cell lines (Fig. 2c and d). In addition, wound healing assay showed that FOXG1 further enhanced the migratory speed of HCC cells (Fig. 2e).

### Overexpression of FOXG1 enhances metastasis of HCC cells in vivo

An orthotopic xenograft tumor model was performed to further explore the ability of FOXG1 to promote metastasis and invasion in HCC cells in vivo. The Huh7/FOXG1 cells and their corresponding vector control cells were injected in the tail vein of nude mice. Strikingly, mice subjected to Huh7/FOXG1 tumors cells displayed prominent lung metastasis, whereas a much lower level of metastasis was found in mice transplanted with control Huh7/vector cells (Fig. 3a and b). Also, H&E staining further confirmed the more pronounced lung metastasis in the FOXG1 group (Fig. 3d). Notably, ectopic FOXG1 expression only decreased the weight of mice in the later stage of experiment (Fig. 3c).

**Fig. 3:** FOXG1 enhances metastasis of HCC cell lines in vivo. **a** Representative bright-field image of the lungs. On day 35, mice that received Huh7/vector or Huh7/FOXG1 cells were anesthetized and sacrificed, and the lungs were collected. Arrows indicate surface metastatic nodules. **b** Number of visible surface metastatic lesions in mice (*n* = 5 per group) that received tail vein injection of Huh7/vector or Huh7/FOXG1 cells. **c** Body weight of BALB/C mice that received transplants of Huh7/vector or Huh7/FOXG1 cells. **d** Lung metastases in mice implanted with Huh7/vector or Huh7/FOXG1 cells were confirmed by hematoxylin and eosin (H&E) staining

The article "Forkhead box (FOX) G1 promotes hepatocellular carcinoma epithelial-Mesenchymal transition by activating Wnt signal through forming T-cell factor-4/Beta-catenin/FOXG1 complex" was retracted in 2023. Reasons: duplicated images; original data or images not available; unreliable data; lack of ethics approval or compliance.

### FOXG1 is essential for EMT characteristics in HCC cells

It is yet to be proven whether FOXG1 is merely a physical marker of EMT or it also contributes to the traits of the progressive phenotype. Therefore, we performed FOXG1 knockdown experiment using a retroviral-based approach in Huh7 and PLC/PRF5y cells. After confirming that 70–80% of FOXG1 were knocked down successfully, we found the elevation of E-cadherin expression in epithelial markers, and the decrease of vimentin and fibronectin levels in mesenchymal markers by Western blotting (Fig. 4a) and Immunofluorescence (Fig. 4b) analysis. The knockdown of FOXG1 markedly weakened the invasive capacity of Huh7 and PLC/PRF5y cells, as determined by transwell assay (Fig. 4c and d).

**Fig. 4:** FOXG1 is essential for EMT in HCC. **a** Western blotting analysis and **b** Immunofluorescence analysis of expression of epithelial cell markers (E-cadherin and α-catenin) and mesenchymal cell markers (vimentin and fibronectin) in indicated cells. GAPDH was used as a loading control. **c** Representative migrating images of the indicated Huh7 and PLC/PRF5y cells on uncoated Transwell devices in five random fields. **d** Quantification of the invading cells of the indicated Huh7 and PLC/PRF5y cells on Matrigel-coated Transwell devices in five random fields. Values represent mean ± SD. *P < 0.05. **e** Representative micrographs of wound healing assay of the indicated Huh7 and PLC/PRF5y cells. Wound closures were photographed at 0, 24, and 36 h after wounding. All experiments were repeated at least three times with similar results

### FOXG1 levels correlate with the activation of Wnt/β-catenin signaling in HCC

We used the TOPFlash reporter to ascertain whether FOXG1 affected the transcriptional activity of β-catenin-TCF/LEF. As we expected, TOP/FOP flash assays revealed that overexpression of FOXG1 significantly increased the transcriptional activation of TCF/LEF in Huh7 and PLC/PRF5y cells, whereas knockdown of FOXG1 attenuated the transcriptional activation of TCF/LEF (Fig. 5a). Furthermore, qPCR analysis revealed that FOXG1 overloading increased the mRNA levels of downstream target genes of the Wnt/β-catenin signaling pathway, including c-Myc, Twist, Snail, MMP7, and Bmp4 (Fig. 5b), whereas silencing FOXG1 did the opposite. Overall, these findings suggest that overexpression of FOXG1 can activate the Wnt/β-catenin signaling pathway.

The article "Forkhead box (FOX) G1 promotes hepatocellular carcinoma epithelial-Mesenchymal transition by activating Wnt signal through forming T-cell factor-4/Beta-catenin/FOXG1 complex" was retracted in 2023. Reasons: duplicated images; original data or images not available; unreliable data; lack of ethics approval or compliance.

**Fig. 5:** FOXG1 activates Wnt/β-catenin signaling by inducing nuclear translocation of β-catenin. **a** Huh7 and PLC/PRF5y cells transfected with TOP Flash or FOP Flash, Renilla pRL-TK plasmids and ectopically expressed FOXG1 were subjected to dual-luciferase assays 48 h after transfection. Reporter activity was normalized to Renilla luciferase activity. The group of cells transfected with vector was used as controls. **b** qPCR detection of altered expression of Wnt signal-pathway genes after ectopic FOXG1 expression in the indicated cells. The group of cells transfected with vector was used as controls. **c** Altered nuclear levels of β-catenin and FOXG1 in response to down-regulated FOXG1 expression were detected by western blotting. P84 were used as a loading controls. **d** HCC cells were stained with fluorescent antibodies against β-catenin (red) or FOXG1 (green) and nuclei were counterstained with DAPI (blue). Representative confocal immunofluorescence images are shown

### FOXG1 mediated β-catenin nuclear translocation by direct binding in vitro

It is well established that nuclear translocation of β-catenin is associated with Wnt signal activation. We wondered whether FOXG1 plays a role in β-catenin nuclear localization. Western blotting analysis of nuclear fraction showed that down-regulation of FOXG1 reduced nuclear β-catenin levels (Fig. 5c), while up-regulated FOXG1 increased its expression (Fig. 5d). Likewise, the immunofluorescence confirmed these results (Fig. 5e).

Since FOXG1 can bind to proteins and act as a molecular chaperone, we hypothesized that the function of FOXG1 protein binding was related to the promotion of nuclear translocation of β-catenin. Therefore, the interaction between β-catenin and FOXG1 was tested by IP analysis in Huh7 HCC cells (Fig. 6a) and 293 T cells transfected with FLAG-tagged β-catenin and FOXG1 (Fig. 6b and c). In a FOXG1 pull-down assay, the purified FLAG-β-catenin bound directly to FOXG1 directly. Reciprocally, in an IP assay using an anti-FLAG antibody, FOXG1 also bound to FLAG-β-catenin. It implies that FOXG1 could function by directly binding to β-catenin.

**Fig. 6:** FOXG1 binds directly to β-catenin. **a** Immunoprecipitation (IP) assay detected the binding of endogenous FOXG1 and β-catenin. **b** IP assay detected the binding of exogenous FOXG1 and β-catenin using anti-FOXG1 to pull down, and followed by immunoblotting (IB) with anti-FLAGantibody. **c** IP assay detected the binding of exogenous FOXG1 and β-catenin using anti-FLAG-β-catenin to pull down and followed by immunoblotting (IB) with anti-FOXG1. **d** Schematic representation of FLAG-tagged full-size and mutant β-catenin. NH2- (gray) and COOH-terminal (black) domains and the 12 internal armadillo-like repeats of β-catenin are indicated. Six different stretches of unrepeated amino acid deletions of β-catenin and the full-size β-catenin are shown in rows 1–7. Twelve internal armadillo-like repeats are shown as numbered boxes. The positions of the amino acid sequences shown and FOXG1 binding ability appear at right. **e** Protein lysates were immunoprecipitated with FLAG anti serum. Equivalent fractions of the immunoprecipitates were separated by SDS-PAGE and blotted with the indicated monoclonal antibodies to analyze binding of mutant β-catenin to FOXG1

As showed in Fig. 6d, β-catenin consists of an NH2-terminal domain (residues 1–110), a central armadillo (Arm) repeat domain (residues 141–664) composed of 12 Arm repeats and a COOH-terminal domain (residues 625–782). Using a series of bacterially expressed GST-β-catenin deletion mutant proteins, we found that Arm repeats 3–5 of β-catenin bound to FOXG1 (Fig. 6e).

The article "Forkhead box (FOX) G1 promotes hepatocellular carcinoma epithelial-Mesenchymal transition by activating Wnt signal through forming T-cell factor-4/Beta-catenin/FOXG1 complex" was retracted in 2023. Reasons: duplicated images; original data or images not available; unreliable data; lack of ethics approval or compliance.

### Mutual recruitment of FOXG1 and β-catenin to Wnt target-gene promoters

Because the FOXG1-β-catenin complex could activate target genes for the Wnt pathway, we speculate that FOXG1 might bind to TCF4, which is a well-known binding partner and target for transcription of β-catenin. Therefore, 293 T cells transfected with FLAG-tagged FOXG1 and myc-tagged TCF were detected by IP to explore the interaction between TCF and FOXG1. In a myc-TCF pull-down assay, purified FLAG-FOXG1 bound to TCF directly (Fig. 7a). And TCF also bound to FLAG-FOXG in an IP assay using an anti-FLAG antibody (Fig. 7b). To distinguish the role of FOXG1 as a β-catenin binding partner and the possibility of FOXG1 as a DNA binding transcription factor, we generated the TCF4 dominant negative mutant (TCF4 DN), which is incapable of β-catenin binding. As with the FOXG1 overexpression, constitutively stabilized β-catenin continued to activate TOP Flash, which is inhibited by TCF4 siRNA in HCC cells (Fig. 7c). Conversely, TCF4 DN, which could not bind to β-catenin, abolished the activation of TOPFlash by FOXG1 (Fig. 7c), suggesting that the effect of FOXG1 is mediated by binding of β-catenin to TCF4.

**Fig. 7:** FOXG1 is a TCF4 binding partner that enhances TCF4 activity. **a** Lysates of 293FT cells expressed myc-TCF4 and FLAG-FOXG1, or a control vector subjected to IP using anti–myc-TCF4 (Upper panel) and anti-FLAG-FOXG1 (lower panel**)** antibodies, followed by IB with anti-myc or anti-FLAG antibody. **b** Mutual dependence of FOXG1 and TCF4 in activating the TOP Flash reporter. FOP Flash was used as negative control. 293 T cells were cotransfected with FOXG1 expression plasmid, TCF4 siRNA, TCF dominant negative (TCF4 DN) expression plasmid, and TCF4-siRNA alone or in combination as indicated. Values are mean ± SD of triplicate samples. **c** ChIP assays of Wnt responsive enhancers (WREs) in the LEF-1 promoter or the ORF region of the LEF-1 gene were performed in Huh7 cells. **d** ChIP assays were performed in Huh7 cells transfected with FOXG1-siRNA (top), β-catenin-siRNA (middle), and TCF4-siRNA or control siRNA (bottom). **e** Lysates of 293FT cells expressing FLAG-FOXG1 and myc-TCF4 with or without β-catenin co-transfection were subjected to IP using anti-FOXG1 or anti-TCF4 antibodies, followed by IB with anti-myc or anti-FLAG antibodies. **f** Lysates of 293FT cells expressed FOXG1 and FLAG-β-catenin with or without myc-TCF4 co-transfection were subjected to IP using anti-FOXG1 or anti-β-catenin antibodies, followed by IB with anti-FLAG or anti-FOXG1 antibody

Another hypothesis to be tested is that FOXG1 might be recruited to TCF/LEF binding elements (TBEs)/WREs in chromatin. The results showed that overexpression of FOXG1 in 293 T cells increased the activity of the LEF-1 promoter (Fig. 7d). And the depletion of FOXG1 diminished the binding of β-catenin to the LEF-1 promoter (Fig. 7e). Moreover, siRNA-mediated depletion of β-catenin reduced the association of FOXG1 and LEF-1 (Fig. 7e), indicating that the association of FOXG1 with LEF-1 is mediated by β-catenin.

The article "Forkhead box (FOX) G1 promotes hepatocellular carcinoma epithelial-Mesenchymal transition by activating Wnt signal through forming T-cell factor-4/Beta-catenin/FOXG1 complex" was retracted in 2023. Reasons: duplicated images; original data or images not available; unreliable data; lack of ethics approval or compliance.

In addition, the association of β-catenin or FOXG1 with the LEF-1 promoter diminished upon the depletion of TCF4 (Fig. 7e). By using the exogenous Myc-TCF4 and FLAG-FOXG1 or FLAG-β-catenin, we found that the binding of FOXG1 and TCF4 was decreased upon β-catenin depletion (Fig. 7f), whereas the binding of FOXG1 and β-catenin remained unchanged when TCF4 was depleted (Fig. 7g). The above results indicate that FOXG1 and β-catenin are mutually dependent for recruitment to WREs occupied by TCF4 in Wnt target-gene promoters.

### FOXG1 expression correlates with activation of Wnt/β-catenin signaling in HCC

IHC analysis was used to examine whether the FOXG1/β-catenin/TCF axes identified in HCC cells were clinically relevant. As shown in Fig. 8a, HCC tissue with a higher FOXG1 expression level also showed the higher expression levels of TCF4 and β-catenin. Conversely, the lower FOXG1 expression level is accompanied with the lower expression of the latter two. And the analysis of IHC scores also confirms this finding (*P* < 0.05) (Fig. 8b). The expression of FOXG1 was positively correlated with that of TCF4 (*P* = 0.048, R2 = 0.505) and β-catenin (*P* = 0.021, R2 = 0.515) (Fig. 8c). In general, up-regulated FOXG1 is closely related to with the expression of β-catenin and TCF4, which in turn activates the Wnt/β-catenin signaling pathway to enhance the metastasis of HCC cells.

The article "Forkhead box (FOX) G1 promotes hepatocellular carcinoma epithelial-Mesenchymal transition by activating Wnt signal through forming T-cell factor-4/Beta-catenin/FOXG1 complex" was retracted in 2023. Reasons: duplicated images; original data or images not available; unreliable data; lack of ethics approval or compliance.

**Fig. 8:** FOXG1 expression correlates with Wnt/β-catenin pathway activation in human HCC. **a** Tissue microarray of IHC showing that TCF4 and β-catenin expression levels were associated with FOXG1 expression in the 105 primary human HCC specimens with or without metastasis. Two representative cases are shown. **b** Percentages of the 105 primary human HCC specimens showing low or high TCF4 and β-catenin protein expression detected by IHC, relative to low/high FOXG1 expression. **c** Correlation analysis of FOXG1 expression with TCF4 (left) and β-catenin (right) expression in 105 HCC samples. Some points represent more than one specimen

## Discussion

In the present study, we provide evidence for a novel mechanistic link between FOXG1 and the oncogenic Wnt/β-catenin signaling pathway in HCC. We found that FOXG1 was significantly up-regulated in HCC and was positively correlated with poor prognosis. Overexpression of FOXG1 promotes the metastasis and invasion of HCC in vitro or in vivo, while the down-regulation of Foxg1 inhibits these occurrences. Furthermore, we demonstrated that FOXG1 could activate the Wnt/β-catenin pathway by directly stimulating β-catenin nuclear translocation through binding β-catenin and TCF4. It implies that FOXG1 plays a role as an oncogene in HCC and may be an important target for clinical intervention.

FOXG1, as a member of FOX gene superfamily, has been revealed to play an important role in embryogenesis and cancers. Other members of this superfamily, such as FOXKs [13], FOXM1 [14], FOXQ1 [22], FOXP3 [23], FOXF2 [24], FOXO1 [25], FOXR2 [26], FOXA2 [27] and FOXL1 [28], have all been shown to interact with β-catenin and play a role in the EMT of cancer cells. Recent studies found that FOXG1 is frequently overexpressed in different types of human tumors as well, including ovarian cancer [29], bladder carcinoma [30], glioblastoma [31] and hepatoblastoma [32]. For example, FOXG1 has been shown to be a prognostic predictor of bladder carcinoma and its expression level correlated with the stage of ovarian cancer [29, 30]. Among 16 cases of hepatoblastoma, 13 cases showed the increased copy of FOXG1, and expression level was negatively correlated with p21 expression level [32]. But such an oncogenic function of FOXG1 and the relationship with the Wnt signaling pathway in HCC remained unclear. We found that overexpression of FOXG1 in HCC cells promoted the EMT phenotype, whereas silencing FOXG1 inhibited it. These results suggest that up-regulation of FOXG1 enhances tumorigenicity and promotes EMT in HCC cells, which may hold promise for development of novel therapeutic treatments to prevent metastasis.

The article "Forkhead box (FOX) G1 promotes hepatocellular carcinoma epithelial-Mesenchymal transition by activating Wnt signal through forming T-cell factor-4/Beta-catenin/FOXG1 complex" was retracted in 2023. Reasons: duplicated images; original data or images not available; unreliable data; lack of ethics approval or compliance.

Aberrant activation of the Wnt/β-catenin signaling pathway is commonly found in many types of human cancers and is thought to promote tumor progression [9]. Multiple key regulators, such as β-catenin, GSK-3β, APC, and TCF/LEF, have been found to be ectopically expressed in HCC, which contributes to the promotion of tumor progression through regulation of the oncogenic Wnt/β-catenin pathway [33]. Nuclear translocation of β-catenin and transcriptional activation of downstream TCF/LEF target genes are the core events of Wnt/β-catenin signaling pathway. Although several mechanisms have been proposed, the molecular mechanisms of β-catenin nuclear translocation and activation remain enigmatic [34, 35]. Consistently, we found that the Wnt/β-catenin pathway was hyperactivated in human HCC cell lines. Moreover, we confirmed that FOXG1 directly binds to and positively regulates β-catenin, which in turn promotes β-catenin nuclear translocation, induces transcriptional activation of TCF/LEF and up-regulates numerous Wnt/β-catenin downstream genes. Overall, these results reveal a novel molecular mechanism underlying the hyperactivation of Wnt/β-catenin pathway in HCC and suggest that FOXG1/β-catenin/TCF4 are potential targets for HCC drug therapy.

Additionally, JASPAR database analysis showed that the FOXG1 promoter contains a NF-κB and MET-specific binding site. In HCC, close to 80% of patients develop tumors against a background of chronic liver inflammation. However, little is known about the specific molecular mechanisms underlying this process. As confirmed the activation of NF-κβ mediates liver oncogenes in mice, the lymphotoxin is over-expressed in a liver-specific manner [36]. Mice in this model developed chronic hepatitis, followed by HCC, at the age of 12 months. Whether NF-κB participates in the activation of FOXG1-mediated Wnt-pathway to enhance the tumor-forming capability of HCC cells deserves further investigation. Furthermore, it has been reported that β-catenin and HGF-mediated signaling pathways cooperate in hepatocyte proliferation, which may be crucial in liver development, regeneration following partial hepatectomy and the pathogenesis of HCC. It also deserves further study whether the pro-inflammatory microenvironment induced by NF-κB and hepatocyte growth factor (HGF) can sustain the FOXG1/Wnt activation to promote tumorigenicity and the EMT phenotype of HCC.

The article "Forkhead box (FOX) G1 promotes hepatocellular carcinoma epithelial-Mesenchymal transition by activating Wnt signal through forming T-cell factor-4/Beta-catenin/FOXG1 complex" was retracted in 2023. Reasons: duplicated images; original data or images not available; unreliable data; lack of ethics approval or compliance.

## Conclusions

In summary, the present study demonstrated that FOXG1 promotes tumor growth in HCC. The up-regulation of FOXG1 dramatically promoted EMT of HCC cells by inducing nuclear shuttle of β-catenin and consequently retains it in the nucleus. In the nucleus, FOXG1/β-catenin complex binds to TCF4 and enhances its transcriptional activity. These findings reveal a novel mechanism of hyperactivation of the Wnt/β-catenin signaling pathway in HCC, suggesting that FOXG1 might activate that pathway through multiple mechanisms by inhibiting β-catenin degradation, accumulating nuclear β-catenin levels and increasing TCF4 transcriptional activity. More broadly, FOXG1 may serve as a potential therapeutic target for HCC.

## Supplementary information

**Additional file 1: Table S1.** Clinicopathological Characteristics of Clinical Samples and Expression of FOXG1 in HCC. **Table S2.** Correlation between FOXG1 Expression and Clinico-pathologic. (DOCX 24 kb)

**Additional file 2.** Supplemental material and methods. (DOCX 23 kb)

## Data Availability

All data generated or analysed during this study are included in this published article and its supplementary information files.

## Abbreviations

AFP: α-fetoprotein
ANT: adjacent nontumor tissue
ChIP-qPCR: Chromatin immunoprecipitation-qPCR
CIRR: cirrhotic liver tissue
EMT: epithelial-mesenchymal transition
FOX: Forkhead Box
HBV: hepatitis B virus
HCC: hepatocellular carcinoma
HGF: hepatocyte growth factor
IF: Immunofluorescence
IHC: Immunohistochemistry
IP: Immunoprecipitation
LEF/TCFs: lymphoid enhancer factor/T cell factor proteins
WREs: Wnt responsive enhancers
